The article "Comprehensive Analysis of Differently Expressed and Methylated Genes in Preeclampsia" was published in 2020. Journal: Comput Math Methods Med.

# Comprehensive Analysis of Differently Expressed and Methylated Genes in Preeclampsia

**DOI:** 10.1155/2020/2139270

**Published:** 2020-11-01

**Authors:** Wenyi Xu, Ping Ru, Zhuorong Gu, Ruoxi Zhang, Xixia Pang, Yi Huang, Zhou Liu, Ming Liu

**Affiliations:** ^1^Department of Obstetrics and Gynecology, Tongren Hospital, Shanghai Jiao Tong University School of Medicine, Shanghai 200032, China; ^2^Department of Obstetrics and Gynecology, Kongjiang Hospital, Shanghai 200093, China; ^3^Department of Life Science, Sichuan Agricultural University, Sichuan 625014, China; ^4^Department of Health Sciences Affiliated Zhoupu Hospital, Shanghai University of Medicine, Shanghai 200032, China

## Abstract

Preeclampsia (PE) is one of the mainly caused maternal and infant incidences and mortalities worldwide. However, the mechanisms underlying PE remained largely unclear. The present study identified 1716 high expressions of gene and 2705 low expressions of gene using GSE60438 database, and identified 7087 hypermethylated and 15120 hypomethylated genes in preeclampsia using GSE100197. Finally, 536 upregulated genes with hypomethylation and 322 downregulated genes with hypermethylation were for the first time revealed in PE. Gene Ontology (GO) analysis revealed that these genes were associated with peptidyl-tyrosine phosphorylation, skeletal system development, leukocyte migration, transcription regulation, T cell receptor and IFN-*γ*-involved pathways, innate immune response, signal transduction, cell adhesion, angiogenesis, and hemopoiesis. Kyoto Encyclopedia of Genes and Genomes (KEGG) pathway analysis demonstrated that aberrantly methylated differentially expressed genes were involved in regulating adherens junction, pluripotency of stem cell regulation, immune processing, T cell receptor and NF-*κ*B pathways, HTLV-I and HSV infections, leishmaniasis, and NK-induced cytotoxicity. Protein-protein interaction (PPI) network analysis identified several hub networks and key genes, including MAPK8, CCNF, CDC23, ABL1, NF1, UBE2E3, CD44, and PIK3R1. We hope these findings will draw more attention to these hub genes in future PE studies.

## 1. Background

As a kind of pregnancy-induced hypertension, preeclampsia (PE) is one of the mainly caused maternal and infant incidences and mortalities worldwide [1, 2]. Numerous body organs and functional systems could be affected by PE, followed by emerging renal failure, ischemic heart, type II diabetes, etc. [1–3]. Several researches have shown a part of external and internal factors that had been identified to induce PE [4]. Currently, trophoblast invasion and failure of spiral artery transformation have been considered to be one inducer of PE [5]. Even though perinatal care was improved, the ratio occurrence of PE has not been reduced [6, 7]. Up to date, the inherent mechanism of PE taken part in many physiological disorders stayed elusive.

The article "Comprehensive Analysis of Differently Expressed and Methylated Genes in Preeclampsia" was published in 2020. Journal: Comput Math Methods Med.

Many studies have identified a large number of differentially expressed genes (DEGs) and differentially methylated genes (DMGs) in PE based on advanced technologies [8–12]. Liu et al. reported that 268 dysfunctional genes were identified in PE, which were related to hormone activity and immune response. Besides, this study revealed TLR2, GSTO1, and mapk13 functioned importantly in the progression of PE [10, 11]. Presently, no studies to investigate the regulated role of gene expression implicated in PE.

Epigenetics indicated that the change of gene expression was heritable, but did not turn out to be in DNA [13, 14]. Among them, DNA methylation was the mostly generated modification in biological metabolism [15]. DNA methyltransferases (DNMTs) were responsible for transmitting DNA methylation to target sites [16]. Nevertheless, the details towards the methylation are not fully understood.

Here, we wanted to explore the association of gene expression with DNA methylation and potential signal pathway in PE development. Therefore, we evaluated the unknown interaction and related signaling pathways of DEG and DMGs in PE by gene expression microarray data (GSE60438) [12] and gene methylation microarray data (GSE100197) [17]. To this end, we attempted to uncover the potential indicator for early diagnosis and prognosis of PE, and also give a hint of probing the involved pathways of DEG/DMGs in PE.

## 2. Materials and Methods

### 2.1. Microarray Data

Differently expressed genes (DEGs)/differently methylated genes (DMGs) were individually analyzed by GSE60438 [12] (including 47 preeclampsia and 48 normal samples) and GSE100197 (including 22 preeclampsia and 51 normal samples) [17]. The details could be seen in the website https://www.ncbi.nlm.nih.gov/geo/.

### 2.2. Data Processing

GEO2R is an online tool that allows users to perform comparisons between different groups in GEO series, which depends on the GEOquery and the Linear Models for Microarray Analysis (LIMMA) R packages [18, 19]. The raw data in TXT format were checked in Venn software online to detect the commonly DEGs among the three datasets. The cutoff standards of DEGs were defined as *P* < 0.05 and fold change > 2, while those of DMGs were indicated as FDR < 0.05 and a fold change > 2.

### 2.3. The Gene Ontology (GO) and Kyoto Encyclopedia of Genes and Genomes (KEGG) Pathway Analysis

DAVID [20] was conducted to do bioinformatics analysis. Significant difference was indicated as *P* < 0.01.

The article "Comprehensive Analysis of Differently Expressed and Methylated Genes in Preeclampsia" was published in 2020. Journal: Comput Math Methods Med.

### 2.4. Construction of Protein-Protein Interaction (PPI) Network

PPI network, including highly methylated and lowly methylated genes, was constructed by STRING database. Interaction score of 0.4 was regarded as cutoff. Cytoscape and the Molecular Complex Detection (MCODE) algorithm were separately applied to visualize PPI network and screen modules. The Molecular Complex Detection (MCODE) app was used to analyze PPI network modules [21], and MCODE scores > 3 and the number of nodes > 5 were set as cutoff criteria with the default parameters (degree cutoff ≥ 2, node score cutoff ≥ 2, K‐core ≥ 2, and max depth = 100). DAVID was utilized to perform pathway enrichment analysis of gene modules. Finally, cytoHubba, a Cytoscape plugin, was utilized to explore PPI network hub genes; it provides a user-friendly interface to explore important nodes in biological networks and computes using eleven methods, of which MCC has a better performance in the PPI network [22].

## 3. Results

### 3.1. Identification of Aberrantly Methylated DEGs in PE

After microarray analysis, our data have shown upregulated and downregulated 3378 DEGs which were 1663 and 1715, respectively. We identified 7087 highly methylated and 15120 lowly methylated genes in PE after relative to normal samples. 829 highly methylated genes (Figure 1(c)) with enhanced level and 408 lowly methylated genes (Figure 1(d)) with weak level were classified after overlapping DEGs and aberrantly methylated genes.  Figure 1(a) shows DEGs in GSE60438 and Figure 1(b) illustrates DMGs of PE and normal tissue. The top 10 upregulated and downregulated genes in PE are shown in Tables 1 and 2.

### 3.2. Functional Analysis

GO analysis indicated that high methylation of genes with increasing expression was generally concentrated in peptidyl-tyrosine phosphorylation, skeletal system development, regulation of bone resorption, mitotic cell cycle, peptidyl-serine phosphorylation pathway, movement of cell or subcellular component, axonogenesis, retina layer formation, calcium ion homeostasis, and cell proliferation (Figure 2(a)).

Low methylation of genes with reduced expression was abounded in leukocyte migration, transcription regulation, T cell receptor and IFN-*γ*-involved pathways, innate immune response, signal transduction, cell adhesion, angiogenesis, and hemopoiesis (Figure 2(b)).

### 3.3. Analysis of Pathway

Upregulated genes with high methylation were dramatically enriched in adherens junction, pluripotency of stem cell regulation, proteoglycans in cancer, the ErbB and sphingolipid signaling pathways, actin cytoskeleton process, ovarian steroidogenesis, carbon metabolism, renal carcinoma, and metabolic pathways (Figure 3(a)).

The article "Comprehensive Analysis of Differently Expressed and Methylated Genes in Preeclampsia" was published in 2020. Journal: Comput Math Methods Med.

Downregulated genes with hypermethylation were enriched in cell adhesion, immune processing, T cell receptor and NF-*κ*B pathways, HTLV-I and HSV infection, leishmaniasis, and NK-induced cytotoxicity (Figure 3(b)).

### 3.4. PPI Network Establishment and cytoHubba Analysis

For strong expression of genes with hypomethylation, 264 nodes and 456 edges were elected. For weak expression of genes with hypermethylation, 159 nodes and 290 edges were obtained (Figure 4). For upregulated oncogenes with hypomethylation, 380 nodes and 1170 edges are shown in Figures 4 and 5. Downregulated TSGs with hypermethylation are indicated in (Figure 5). Totally, 212 nodes and 458 edges were included in TSGs. MCODE plugin detection revealed that FLNA and PRKCB were reduced with hypermethylation, and AKT1, PRDM10, CCND1, and FASN 4 were heightened with hypomethylation.

### 3.5. Key Module and Gene Analysis

There is obvious difference between three modules with hypomethylation of upregulated genes and three modules with hypermethylation of downregulated genes (Figure 4). The hub network 1 of overexpressed hypomethylated genes included CCNF, RNF14, UBE2B, SH3RF1, UBE2V1, FBXO30, FBXW7, FBXO17, PJA2, UBE2M, TRIM36, HECW2, UBE2E3, SOCS1, MYLIP, and CDC23. The hub network 2 of overexpressed hypomethylated genes included GPER1, OPN4, GPR17, PLCB4, MCHR2, MCHR1, TAS2R14, PTGER3, CCL4, NPS, KISS1, and ADCY8. The hub network 3 of overexpressed hypomethylated genes included SEC22B, LHB, CGA, HNRNPA3, NEIL3, TAAR6, SLC30A5, GOLIM4, BAG4, ABCB1, GOLGA5, MAN1A2, CRH, PTPN6, PREB, SEC24B, FOLR1, DEPDC1B, TPX2, SLC30A2, CEP152, FGFR1, SGOL2, LIMK1, PSG3, CDC25C, KHSRP, DHX9, SYNCRIP, PAK4, ERBB2, SDC3, SDC1, PSG6, JUP, DCTN3, RPL22L1, KRT19, NUF2, PSG11, NCAPG, QPCT, RHOBTB1, RPL34, SRP19, YWHAE, MATR3, NTF3, LMAN1, PSG4, ERBB3, SPCS3, SEC11A, ARHGEF11, SLC30A1, SLC39A1, TROAP, MAN1C1, MAP2K1, RRAS2, AKT3, SLC39A8, PSG9, TRIP13, TIMP2, TRIM24, and PSG1.

The hub network 1 of downregulated hypermethylated genes included ATG7, UBA7, RNF213, ARIH2, FBXL19, FBXO44, HERC4, and ASB15. The hub network 2 of downregulated hypermethylated genes included SRSF4, RBM5, PRPF3, SF3B1, HNRNPU, CPSF2, and CSTF3. The hub network 3 of downregulated hypermethylated genes included ADCY7, ZAP70, GPR18, LY9, NPBWR1, CD4, ITGA4, CD44, FPR3, SSTR1, GABBR1, GNB4, CCR3, and SLAMF1 (Figure 5).

Among these genes, MAPK8, CCNF, CDC23, ABL1, NF1, UBE2E3, CD44, and PIK3R1 were identified as key regulators in PE by connecting with more than 20 different genes in the network.

## 4. Discussion

Preeclampsia was reported to be largely related to increasing incidence and death of maternal organ, dysfunction of maternal organ, or restricted growth of foetal organ [23]. However, the mechanisms related to this disease remained largely unclear. Emerging studies demonstrated that the aberrant changes in DNA methylation contributed to the abnormal expression of key genes in multiple diseases, such as preeclampsia [24]. Therefore, conclusive delineation of gene level and methylation could provide novel insights to identify novel predictive and therapeutic targets for preeclampsia. The present study identified 1716 high expressions of gene and 2705 low expressions of gene using GSE60438 database, and identified 7087 hypermethylated and 15120 hypomethylated genes in preeclampsia using GSE100197 database. Finally, 536 upregulated genes with hypomethylation and 322 downregulated genes with hypermethylation were for the first time revealed in PE.

The article "Comprehensive Analysis of Differently Expressed and Methylated Genes in Preeclampsia" was published in 2020. Journal: Comput Math Methods Med.

Furthermore, bioinformatics analysis was performed to reveal the potential functions of these aberrantly methylated DEGs in preeclampsia. Meanwhile, we identified aberrantly methylated DEGs in preeclampsia that were associated with transcription level, cell defense, cell immunity response, IFN-*γ*-involved pathway, and T cell receptor pathway. These findings were consistent with previous reports that abnormal regulation of immune functions was related to preeclampsia progression [25]. Our results showed that hypomethylated highly expressed genes were related to the regulation of multiple key signalings in cell biology, such as cell mitosis, axonogenesis, Ca^2+^ homeostasis, cell proliferation, the ErbB signaling pathway, ovarian steroidogenesis, and the sphingolipid signaling pathway. As a second messenger, Ca^2+^ acts as a primary role in cell growth, cell death, etc. [26]. Downstream pathway was activated by Ca^2+^ via exporting intracellular organelles or importing extracellular depots [27–29]. As the foremost form of Ca^2+^ pathway, downstream effectors of intracellular Ca^2+^ oscillations included transcription factors, kinases, and other functional proteins [30–32]. Our data suggests that the imbalance of Ca^2+^ in homeostatic cells may be linked to the progression of PE. A very interesting finding is that a recent study showed that Ca^2+^ signaling is related to the activation of the ErbB pathway, involving lots of tyrosine kinases, and is resistant to radiation and chemotherapy in many tumors. Two tyrosine residues were dimerized and phosphorylated by EGFR after conjugating to ligands [33, 34]. Conversely, these phosphorylated tyrosines could be regarded as binding sites for some signal transmitters which participated in biological pathways.

Moreover, we revealed that hypermethylated genes with low expression were associated with cell adhesion, angiogenesis, hemopoiesis, and the NF-kappa B signaling pathway. A recent study showed that the genes of cell adhesion signaling in the preeclamptic placentas were observed to be differentially methylated [35]. Endothelial cells have been confirmed to be acted as the key inducer to angiogenesis via cell-promoting cell metastasis [36]. Notedly, EPCs (endothelial progenitor cells) functioned importantly in the generation of the postnatal blood vessel and vascular homeostasis [37]. The endothelial dysfunction in PE probably led to the destructive fetoplacental angiogenesis and neovasculogenesis [38]. The decreasing level of some proangiogenic factors in the placenta was observed in the early-stage PE not the late-stage PE [38]. There were more than 2 angiogenesis-related genes with the reduced level in the early-stage PE after comparison with the late-stage PE or control [39]. Currently, our data revealed that the growth/migration of human umbilical vein endothelial cells was suppressed in the early-stage PE compared to that in the late-stage PE or control, suggesting negative regulation of angiogenesis in PE.

The article "Comprehensive Analysis of Differently Expressed and Methylated Genes in Preeclampsia" was published in 2020. Journal: Comput Math Methods Med.

In order to identify the hub genes and networks in PE, we conducted a PPI network analysis. The upregulated hypomethylated PPI network was composed of 380 nodes and 1170 edges, while the downregulated hypermethylated PPI network consisted 380 nodes and 1170 edges. Furthermore, we identified 6 hub networks using MCODE plugin in Cytoscape software. Among these genes, MAPK8, CCNF, CDC23, ABL1, NF1, UBE2E3, CD44, and PIK3R1 were identified as key regulators in PE. MAPK8 belonged to mitogen-activated protein kinase (MAPK) family which is critical for cellular function through regulating numerous signaling pathways [40]. A recent study showed that MAPK8, which is necessary for epithelial-mesenchymal transition, is responsible for regulating transcription [41]. CDC23 is a cell cycle regulator, exhibiting importantly in both initiation and elongation of DNA replication [42, 43]. Loss of NF1 results in dysregulation of MAPK, PI3K, and other signaling cascades, to promote cell proliferation and to inhibit cell apoptosis. UBE2E3 have a key role in regulation of cell aging which was essential for homeostasis of tissues. Cells' absence of UBE2E3 will be senescent even though without DNA damage [44]; meanwhile, accumulated mitochondrial and lysosomal mass and raised basal autophagic flux were shown in UBE2E3 absent cells. CD44 as a member of CAM family mostly takes part in cell movement and proliferation [45]. PIK3R1-encoded PI3K, p85*α*, could conjugate, maintain, and suppress catalytic subunit of PI3K p110 [46]. Not only did mutated PIK3R1 reduce the subtype of P110 inhibition but also destroyed the new regulatory effect of p85*α* on PTEN or activated a new signal pathway.

The article "Comprehensive Analysis of Differently Expressed and Methylated Genes in Preeclampsia" was published in 2020. Journal: Comput Math Methods Med.

Nevertheless, our studies still had some limitations. Firstly, our researches concentrated on the classification of DEG with different methylations. Secondly, our researches should broaden the analysis datasets so as to acquire comprehensive data. Thirdly, we needed to conduct qRT-PCR or western blot to further ensure the selected gene level in PE samples. Finally, the function and mechanism of biomarkers in PE need to be further studied in vivo and in vitro.

## 5. Conclusion

Collectively, we identified some oncogene expression patterns and their links with corresponding pathways in PE, providing a hint of exploring the mechanisms implicated in PE onset and development.

## Figures and Tables

**Figure 1:** Identification of aberrantly methylated differentially expressed genes in PC. (a) Identification of differently expressed genes in PC using GSE60438. (b) Identification of differently methylated genes in PC using GSE100197. (c) A total of 829 upregulated hypomethylated genes were identified in PC. (d) A total of 409 downregulated hypermethylated genes were identified in PC.

**Figure 2:** GO analysis of aberrantly methylated differentially expressed genes in PC. GO analysis of upregulated hypomethylated genes (a) and downregulated hypermethylated genes (b) in PC.

**Figure 3:** KEGG pathway analysis of aberrantly methylated differentially expressed genes in PC. KEGG pathway analysis of upregulated hypomethylated genes (a) and downregulated hypermethylated genes (b) in PC.

**Figure 4:** Protein-protein interaction network analysis of upregulated hypomethylated genes in PC. We constructed PPI networks of upregulated hypomethylated genes in PC.

**Figure 5:** Protein-protein interaction network analysis of downregulated hypermethylated genes in PC. We constructed PPI networks of downregulated hypermethylated genes in PC.

**Table 1:** The top 10 upregulated genes in PE compared to normal samples.

Gene	AVE NC	AVE PE	FC	*P* value
CGB5	7.140694905	8.555772571	2.666740913	0.000524413
CRH	7.35786819	8.743007971	2.611972633	0.00019934
CGB1	7.330520262	8.540119829	2.312734358	0.00097466
KISS1	7.882624452	9.119308971	2.356563438	0.00381749
ADAM12	8.732927738	10.04238443	2.478481844	0.002319055
DLK1	7.393902548	8.500453743	2.153302782	0.010929138
CGA	8.495501333	9.765370743	2.41139737	0.003638636
PSG6	8.514054476	9.723809743	2.312983969	0.007442872
CGB8	7.176896333	8.174694886	1.996950473	0.001320154
PAGE4	7.430149214	8.450650829	2.028624174	0.009079707

**Table 2:** The top 10 downregulated genes in PE compared to normal samples.

Gene	AVE NC	AVE PE	FC	*P* value
LOC647169	8.7158875	8.070096229	0.639142146	0.012472714
FCN1	10.84868995	10.03952706	0.570712911	0.023728745
LYZ	12.23783017	11.29681926	0.520867776	0.002834118
CCL2	10.03269452	9.2354408	0.575443535	0.000263349
CX3CR1	8.787585643	8.068285229	0.607391905	0.007852246
CCL18	8.994379333	8.217637057	0.583683311	0.000247839
GSTA1	8.678950238	7.926187143	0.593465844	0.006579547
PI3	8.461040238	7.713865943	0.595769307	0.013088748
LTB	9.728131619	8.857907943	0.547062027	0.00330664
GSTA1	8.871995429	8.0231716	0.555237214	0.004279029

The article "Comprehensive Analysis of Differently Expressed and Methylated Genes in Preeclampsia" was published in 2020. Journal: Comput Math Methods Med.

## Data Availability

The datasets used during the present study are available from the corresponding author upon reasonable request.
